# The Trend of Burn Injury Patients in Ningbo between 2012 and 2021: A Clinical Study

**DOI:** 10.1155/2022/9969158

**Published:** 2022-08-12

**Authors:** Youfen Fan, Guoying Jin, Yanyan Pan, Shengyong Cui, Jiliang Li, Neng Huang

**Affiliations:** Burn Department, HwaMei Hospital, University of Chinese Academy of Sciences, No. 41 Northwest Street, Haishu District, Ningbo 315010, Zhejiang Province, China

## Abstract

**Objective:**

This study was designed to understand the local changes of burn injuries in recent 10 years, so as to provide reliable reference data and viewpoints for prevention and vigilance of local burn injuries.

**Methods:**

In this study, 184 patients with a burn injury admitted to our hospital from 2012 to 2021 were enrolled and analyzed retrospectively. According to their information in the electronic database, the number of patients with burn injuries and the location of each disaster each year were analyzed, and the age, sex, hospital stay and hospitalization expense of each patient were collected. With 5 years as the boundary, the patients were divided into a 2012–2016 group and a 2017–2021 group and the differences of the two groups in the abovementioned aspects were compared.

**Results:**

During 2012–2021, the incidence rate of burn injuries in men was higher than that in women and workplaces had a higher burn injury rate than residents' homes. Compared with the period of 2012–2016, the number of fires or explosions and the number of patients with a burn injury during 2017–2028 both increased, but there was no significant change in disaster location, male-female ratio, age, average hospital stay, and average hospitalization expense.

**Conclusion:**

In the face of the increasing prevalence of burn injuries, we should strengthen fire-fighting knowledge-related education and fire prevention management and actively explore post-burn injury treatment strategies and potential treatment targets to promote the development of burn injury management and treatment strategies.

## 1. Introduction

Dust explosion, gas leakage, and boiler explosion often trigger regional fire and result in severe burn injuries to personnel. Burn injuries can give rise to immune disorders, inflammation, and metabolic disorders, and even multiple organ failure and shock in severe cases [1]. Physical pain caused by burn injuries can result in emotional disorders such as anxiety and depression [2]. According to a retrospective study [3], burn injuries are significantly associated with the incidence rate of individual mental disorders. They also seriously compromise the quality of daily life of patients by triggering heat sensitivity, pain, physical and emotional dysfunction, and others [4]. A prospective study in 2017 has revealed that the physical function and mental health of patients decrease significantly within 12 months after burn injuries [5]. Statistics showed that the mortality of burn injuries in China in 2013 was 0.88 per 100,000 people, and the death mostly occurred in the population group of 70 years old and above [6]. As the primary cause of morbidity and disability, burn injuries require long-term care and treatment, bringing huge social and economic burden [7]. Accordingly, burn injuries are a serious public health problem.

Epidemiology reveals the number of sick people, promotes the awareness of all the factors that determine the occurrence of a disease and the understanding of the trend of the disease over a period of time [8, 9]. In recent ten years, there are still few articles about local burn injuries. Additionally, China is still in the stage of development, with a constantly changing epidemic trend of burn injuries, so most of the epidemiology of burn injuries in China only investigates the specific types [10]. Therefore, the improvement in the effects of preventive measures on death and deformity entails an epidemiological study based on local inpatients with a burn injury [11].

For the purpose of understanding the local changes of burn injuries in recent 10 years, this study enrolled 184 patients with burn injuries admitted to our hospital from 2012 to 2021, counted the number of patients with it per year and the location of each fire, and collected the age, sex, hospital stay and hospitalization expense of each patient, with the goal of providing reliable reference data and viewpoints for the prevention and vigilance of local burn injuries.

## 2. Methods

### 2.1. Patients with Burn Injury

The clinical symptoms of all enrolled patients were consistent with the definition of burn injuries. Patients who had been treated against burn injuries in local clinics, community health centers or other hospitals before admission, and those complicated with malignant tumors, major diseases of heart, lung, liver, or kidney, or systemic immune diseases were all excluded. This study was approved by the Medical Ethics Committee of our hospital, and every patient signed an informed consent form after being informed of the study. Finally, 184 patients with burn injuries admitted to our hospital from 2012 to 2021 were included, including 135 males and 49 females. The causes of burn injuries of them included dust explosion, cotton-induced fire, boiler explosion, die casting machine explosion, acetylene fire, gas leakage, plastic explosion, foam explosion, etc. For each burn incident, the number of patients involved is three or more.

### 2.2. Data Collection

Patients with burn injuries admitted to our hospital from 2012 to 2021 were enrolled and retrospectively analyzed in this study. According to their information in the electronic database, the number of patients with a burn injury and the location of each disaster each year were analyzed, and the age, sex, hospital stay, and hospitalization expense of each patient were collected. In the present study, with 5 years as the boundary, the patients were divided into a 2012–2016 group and a 2017–2021 group, and the differences of the two groups in the abovementioned aspects were compared.

### 2.3. Quality Control

Two doctors were arranged to inspect and review the data of enrolled patients, and the research data were reviewed and counted by the doctor specializing in data research. The results were also checked and revised by a doctor with rich experience in epidemiological research. The study was approved by the Human Ethics Committee of the HwaMei Hospital, University of Chinese Academy of Sciences (SL-NBEY-KY-2022-082-01) and conformed to the relevant regulatory guidelines of the national ministries and commissions and CFDA and the ethical principles of the Declaration of Helsinki.

### 2.4. Statistical Analyses

The measurement data were expressed as mean ± standard deviation and compared using the independent-samples *T* test. The counting data were expressed as the number of cases (percentage) and analyzed using the Chi-square test. All tests were two-tailed *t* tests. *P* < 0.05 is considered statistically significant (confidence interval is 95%). GraphPad 9.0 was used to visualize the data into figures, and SPSS22.0 was used to statistically analyze the research data. These data passed the normality test based on the Shapiro–Wilk test before the independent-samples *t* test.

## 3. Results

### 3.1. Number of Fires and Number of Patients with Burn Injury during 2012–2016 and during 2018–2021

In this study, the number of fires and number of patients with a burn injury each year between 2012 and 2021 were counted. As shown in Figure 1, there were 44 fires during 2012–2021, including 15 during 2012–2016 and 29 during 2017–2021, and the number of fires in the last five years increased. As shown in Figure 2, there were 55 patients with a burn injury during 2012–2016 and 129 patients with it during 2017–2021, and the number of them also increased in the last five years.

### 3.2. Fire Places during 2012–2017 and during 2018–2020

In this study, the locations of fires during 2012–2021 were counted, and the changes of fire locations during 2012–2016 and during 2017–2021 were compared. As shown in Table 1, there were 15 fires during 2012–2016, including 10 (66.67%) fires in workplaces (chemical plants, quilt processing plants, food processing plants, textile factories, chemical fiber factories, waste stations, etc.), and 5 (33.33%) fires at homes, and there were 33 fires during 2017–2021, including 24 (72.73%) in workplaces and 9 (27.27%) at homes. The workplaces are still the most common fire places in both the first five years and the last five years, However, there was no significant difference in the fire rate in the workplaces and homes between the two five years.

### 3.3. Gender of Burn Injury Groups during 2012–2016 and during 2018–2020

During 2012–2016, there were 39 (70.91%) males with burn injuries and 16 (29.09%) females with it. During 2017–2021, there were 96 (74.42%) males with burn injuries and 33 (25.58) females with it. During 2012–2016 and 2017–2021, the burn injury rate among males was significantly higher than that among females (Figure 3), but there was no statistical difference in it between the two five years (Table 2).

### 3.4. Burden of Burn Injury-Caused Hospitalization during 2012–2016 and during 2017–2021

The hospitalization burden (average hospital stay and average hospitalization expense) of patients due to burn injury during 2012–2021 was counted as shown in Figure 4. Although the average hospital stay and average hospitalization expense during 2017–2021 increased compared with those during 2012–2016, the difference was not statistically significant.

### 3.5. Statistics on the Age of Patients with Burn Injury during 2012–2016 and during 2017–2020

The ages of patients with a burn injury from 2012 to 2021 was counted, and the average ages of them during 2012–2016 and during 2017–2021 were calculated (Figure 5). According to a statistical comparison, there was no significant difference between the average age of patients with a burn injury during 2012–2016 and that during 2017–2021.

## 4. Discussion

Burn injuries are potentially catastrophic [12]. For developing countries, burn injuries are a common type of injury, which may lead to serious morbidity and mortality [13]. Pathologically, it can trigger infection, sepsis, scar hyperplasia, and other complications, which can seriously threaten the health of patients [13–15]. A significant progress has been achieved in the nursing and treatment of burn injuries in recent years [16]. Statistical research on the population of burn injuries is helpful to understand the local epidemic trend and potential harm of burn injuries. This study collected the data of patients with a burn injury between 2012 and 2021 from the electronic database and analyzed the local change trend of burn injuries in recent ten years, with five years as an interval.

First of all, compared with the period of 2012–2016, the number of fires or explosions in the period of 2017–2021 increased, accompanied by a significantly increased number of patients with a burn injury. In fact, the increase in the scale and number of burn injuries has already become a global trend [17]. The increase in the incidence rate of burn injuries may be closely related to social and economic development [18]. With a large population, China is in the stage of development; so, many patients are affected by burn injuries [19]. The increase in the scale and number of individuals with a burn injury also increased the potential pressure of local treatment to some extent. Industrial workers or other workers who may face fire hazards are more susceptible to burn injuries [20]. This study has also confirmed this conclusion. Although there is no obvious deviation between 2012–2016 and 2017–2021 in the cause of burn injuries and the location of disasters (the workplace is still the place where burn injuries are mostly likely to appear), we still need to be aware that workers lack the necessary fire safety knowledge in the process of work and operation.

Second, we found that there were more males with a burn injury than females with it, and this phenomenon had no significant change in the last decade. In most parts of China, males are more susceptible to burn injuries [21–23], which may be due to the fact that there are more males in high-risk jobs. According to the results, working men seem to be the vulnerable group of burn injuries [24]. One thing to be wary of is that most burn injurers in females occur at homes, which also reminds us the necessity to strengthen residents' knowledge education on fire use and fire prevention at home.

It is noticed that the management and treatment strategies of burn injuries still need further development. In the present study, compared with the period of 2012–2016, the average hospital stay and average hospitalization expense of patients with a burn injury during 2017–2021 did not increase significantly, which indicated that the pressure of local burn injury treatment did not fluctuate (although the number of patients with burn injuries increased). This phenomenon also shows that the management and treatment strategies of burn injuries have not achieved significant development in the last ten years. In fact, there are differences between high-income countries and middle-income countries in terms of hospital stay and treatment cost of burn injuries. In recent years, hospital stay in high-income countries has shown a significant downward trend. The heterogeneity of hospital stay and treatment cost between the two kinds of countries may be related to burn injury management and treatment strategies [25]. High-income countries may have more advanced post-burn injury strategies. Therefore, it is required to promote the development of local burn injury management and treatment strategies and strive to lower the cost and economic burden of patients with a burn injury. In addition, it was found that the burns incorporated were all in batches. Due to economic and technological developments, mass burns do occur from time to time. Burns in batch mean the heavy task of treatment, which tests the ability of the hospital and its staff to cope with them. More advanced treatment strategies will also significantly reduce the treatment stress faced by the staff when dealing with batches of burns and will help to contain further deterioration of the patient's condition.

This study still has some limitations. First of all, due to the limited information collected, we have failed to explore the risk factors affecting the postoperative survival outcome of patients with a burn injury in recent ten years, which is expected to be addressed in future research. We will start a longitudinal study to follow up the patients for a long time, and record the complications, cure time and postoperative quality of life of them in detail, so as to explore the risk factors that affect the outcomes of burn injuries. Second, the burn injury cases included in this study are all from patients in our hospital, which can only be used as reference evidence of local burn injury trends but is not enough to help people know more about burn injury-related information in this province or China. Finally, the sample size of this study is limited, so the sample size can be expanded in future research to verify the findings of this study.

To sum up, in the face of the increasing prevalence rate of local burn injuries, we should strengthen the fire prevention knowledge-related education and fire prevention management in factories, restaurants, waste stations, and other workplaces, and also remind the public to pay attention to the fire safety in daily life to prevent gas leakage. We should also carry out more research to explore the post-burn injury treatment strategies and potential treatment targets to promote the development of burn injury management and treatment strategies and strive to lower the treatment cost and economic burden of patients with a burn injury.

## Figures and Tables

**Figure 1:** The number of fires per year from 2012 to 2021 (Total: 184).

**Figure 2:** The number of patients with burn injury per year from 2012 to 2021 (Total: 184).

**Figure 3:** Annual statistics of males and females with burn injury from 2012 to 2021 (Total: 184, male: 135 and female: 49). Gender composition in 2012–2016 and 2017–2021 was analyzed by the Chi-square test.

**Figure 4:** Burden of burn injury-caused hospitalization during 2012–2016 and during 2017–2021 (a) average hospital stay; (b) average hospitalization expense; in 2012–2016, *n* = 55; in 2017–2021, *n* = 129). The comparison was processed by independent sample *t* test.

**Figure 5:** Average age of patients with burn injury during 2012–2016 and 2017–2020 (In 2012–2016, *n* = 55; in 2017–2021, *n* = 129).

**Table 1:** Fire places during 2012–2016 and during 2017–2021.

	2012–2016	2017–2021	*χ* ^2^	*P* value
			0.183	0.669
Workplaces	10	24		
Home	5	9		

**Table 2:** Statistics of the number of males with burn injury and females with it.

	2012–2016 *n* = 55	2017–2021 *n* = 129	*χ* ^2^	*P* value
			0.24	0.62
Male	39	96		
Female	16	33		

## Data Availability

The clinical data used to support the findings of this study are included within the article.
